# *Ficus exasperata* Attenuates Acetaminophen-Induced Hepatic Damage via NF-*κ*B Signaling Mechanism in Experimental Rat Model

**DOI:** 10.1155/2022/6032511

**Published:** 2022-05-24

**Authors:** Babatunde Oluwafemi Adetuyi, Oluwaseun Abraham Adebisi, Oluwatosin Adefunke Adetuyi, Olubanke Olujoke Ogunlana, Pere-Ebi Toloyai, Chukwuebuka Egbuna, Chukwuemelie Zedech Uche, Johra Khan, Obinna Chukwuemeka Uchenna Adumanya, Kingsley C. Patrick-Iwuanyanwu

**Affiliations:** ^1^Department of Natural Sciences, Faculty of Pure and Applied Sciences, Precious Cornerstone University, Ibadan, Oyo State, Nigeria; ^2^Department of Biochemistry, Osun State University, Osogbo, Osun State, Nigeria; ^3^Department of Biochemistry, Covenant University, Ota, Ogun State, Nigeria; ^4^Department of Medical Biochemistry, Delta State University, Abraka, Delta State, Nigeria; ^5^Africa Centre of Excellence in Public Health and Toxicological Research (ACE-PUTOR), Nutritional Biochemistry and Toxicology Unit, University of Port-Harcourt, Rivers State, Nigeria; ^6^Department of Biochemistry, Faculty of Science, University of Port Harcourt, East-West Road, P.M.B. 5323, Port Harcourt, Rivers State, Nigeria; ^7^Department of Medical Biochemistry and Molecular Biology, Faculty of Basic Medical Sciences, University of Nigeria, Enugu Campus, Nigeria; ^8^Department of Medical Laboratory Sciences, College of Applied Medical Sciences, Majmaah University, Majmaah 11952, Saudi Arabia; ^9^Health and Basic Sciences Research Center, Majmaah University, Majmaah 11952, Saudi Arabia; ^10^Department of Biochemistry, University of Agriculture and Environmental Science, Umuagwo, Imo State, Nigeria

## Abstract

*Ficus exasperata* has been used to treat ulcer, diabetes, fever, and a variety of stress-related disorders. Acetaminophen (APAP) overdose is the most common cause of drug-induced acute liver injury. In this study, we evaluated the hepatoprotective effect and antioxidant capacity of ethanolic extract of *F. exasperata* (EFE) on acetaminophen-induced hepatotoxicity in albino rats. Rats were pretreated with EFE (150, 250, 500 mg/kg) and thereafter received 250 mg/kg APA intraperitoneally (i.p.). The normal control group received distilled water, while the negative control group received 250 mg/kg APAP, respectively. Hepatotoxicity and oxidative stress-antioxidant parameters were then assessed. Flavonoids, saponins, steroids, and glycosides, but not phenolics were detected by EFE phytochemical analysis. No mortality was recorded on acute exposure of rats to varying concentrations of APAP after 24 h; however, a dose-dependent increase in severity of convulsion, urination, and hyperactivity was observed. APAP overdose induced high AST, ALT, ALP, and total bilirubin levels in the serum, invoked lipid peroxidation, depleted GSH, decreased CAT, SOD, and GST levels, respectively. Nitric oxide (NO) level, myeloperoxidase activity, TNF-*α*, IL-1*β*, NF-*κ*B, COX-2, MCP-1, and IL-6 were also increased. Importantly, pretreatment of rats with EFE before acetaminophen ameliorated and restored cellular antioxidant status to levels comparable to the control group. Our results show and suggest the hepatoprotective effect of *F. exasperata* and its ability to modulate cellular antioxidant status supports its use in traditional medicine and renders it safe in treating an oxidative stress-induced hepatic injury.

## 1. Introduction

Environmental exposure to xenobiotics and the use of drugs at nontherapeutic doses are among several factors that cause body tissue damage such as liver. Importantly, oxidative stress involving the generation of reactive oxygen species has been involved in tissue damage [1, 2]. Drug-induced liver injury remains a significant clinical problem. APAP toxicity occurs mainly due to an overdose of acetaminophen and may therefore be a significant cause of liver injury worldwide [3]. APAP is metabolized to the reactive metabolite, NAPQI (N-acetyl-p-benzoquinone imine), by the liver CYP 450 enzymes, which depletes glutathione levels, disrupts thiol redox homeostasis and increases oxidative stress injurious to the liver [4, 5]. Although N-acetylcysteine, (NAC), the antioxidant and common panacea for APAP-induced hepatotoxicity, ameliorates the toxic effect, certain side effects may still lead to liver injury in patients, even at a prescribed safe dose [6]. Hence, a safe therapeutic alternative for APAP detoxification is advocated. Nowadays, more attention has been drawn to the use of herbal products as a major part of alternative medicine, and in fact, a good percentage of the world population now depends on naturally derived medicines for the treatment and management of diseases [7–9]. Recent drug therapies are derived from plants and some of them seem to play important roles in hepatocyte regeneration and healing and thus can be used in the management of liver injury and disorders [1].

*Ficus exasperata* is one of such plant-based therapies. The genus *Ficus* belongs to the Mulberry family (Moraceae). *Ficus exasperata* Vahl is commonly known as sandpaper tree (“Ewe Ipin” in Yoruba) and is widely used in all types of vegetation in West Africa and particularly in secondary forest regrowth [10]. In Nigeria, the young leaves of *F. exasperata* are prescribed as a common antiulcer remedy. Moreover, *F. exasperata* possesses various pharmacological actions including antidiabetic, lipid-lowering, and antifungal activities. Mounting evidence reveals that *F. exasperata* leaves exhibit anti-inflammatory, anxiolytic, anticonvulsant, antipyretic, and antimicrobial activity [11–13]. Although recent toxicity studies involving crude, aqueous, and ethanol leaf extract have shown hepatic and renal toxicity at high doses, lower doses may lead to improved hepatocyte regeneration and may not interfere with tubular function and reduce renal failure risk [14].

Particularly, previous studies have reported the anti-inflammatory, analgesic, and antipyretic activities of *Ficus exasperata* leaf extracts [8]. Since modulation of free radical generation, scavenging and anti-inflammatory activities are strategic in the management of liver damage. *Ficus exasperata* is thus suggested to have a hepatoprotective effect. Our aim here is to evaluate the hepatoprotective activity of ethanolic extract of *F. exasperata* leaves against acetaminophen-induced liver damage in rats, as well as assess the liver functioning by determining the liver serum and oxidative stress markers.

## 2. Materials and Methods

### 2.1. Animals

Albino rats (*Rattus norvegicus*) weighing between 91.6 g and 164.3 g were used in this evaluation. These rats were gotten from Ayoola farm house in Ilorin, Kwara State, Nigeria. They were kept under standard conditions (23 ± 2°C) (55 ± 10% humidity) with 12 h light/dark cycle and standard pellet diet provided as well as free access to water during the experimental period. Importantly, the animals were acclimatized to the environment for 2 weeks before the initiation of the experiment. Ethical approval was obtained for the use of animals in the experiment from the Osun State University Ethical Committee on the use of laboratory animals for research.

### 2.2. Chemicals

Acetaminophen, chloroform, and methanol used were obtained from Fam-lab Nigeria Limited, Akure, and Lixok-k chemicals, Akure, respectively. Alanine transaminase (ALT), aspartate transaminase (AST), gamma glutamyltransferase (GGT) and total protein, and bilirubin were obtained from Randox Laboratories Limited, UK.

### 2.3. Plant Source and Identification

*Ficus exasperata* was obtained from the forest near Ikeji-Arakeji, Osun State. Plants were taken to the Department of Agricultural Sciences, Joseph Ayo Babalola University, for identification.

### 2.4. Preparation and Extraction of Crude Plant Extract

*Ficus exasperata* leaves were air-dried for three weeks and blended into powdery form using an industrial blender. Approximately 250 g of *Ficus exasperata* leaf sample was weighed with electronic balancing and soaked in 700 ml ethanol at room temperature for 48 h. The solvent was filtered using Whatman filter paper and stored in the refrigerator until use.

### 2.5. Phytochemical Screening of Plant Extract

Basic phytochemical screening is the method employed to check the presence of certain bioactive compounds in plants, e.g., antraquinone, tannins, saponins, flavonoids, cardiac glycosides, steroids, phenolics, cardenolides, and denolides. The methods are as follows (AOAC [15], Batiha et al. [16]).

#### 2.5.1. Test for Tannins

About 0.2 g of each portion of plants extract was stirred with 5 ml of distilled water and filtered, and 0.1% ferric chloride reagent was added to the filtrate. A blue black green precipitate was taken as evidence for the presence of tannins.

#### 2.5.2. Test for Saponins

The ability of saponins to produce frothing in ethanol solution and red blood cell haemolysis was used as screening test for these compounds. For the frothing test, each plant extract was shaken with water in test tube and frothing that persists on warming was taken as preliminary proof of saponin presence.

#### 2.5.3. Test for Anthraquinone

About 0.2 g of the extract was shaken with 5 ml concentrated benzene and 5 ml of 10% NH_3_ solution. The mixture was shaken and the presence of pink, red, or violet colour in the ammonia phase indicates the presence of anthraquinones.

#### 2.5.4. Test for Flavonoids

One milliliter (1 ml) of 10% NaOH was added to 3 ml of *F. exasperata* ethanol extract. A yellow colour development indicates the presence of flavonoids.

#### 2.5.5. Test for Cardiac Glycosides

About 1 ml of *F. exasperata* ethanol extract was added to 2 ml of chloroform and shaken. The mixture was allowed to settle down, and H_2_SO_4_ was added carefully to calm the solution. A reddish-brown colour at the interface indicates the presence of aglycone portion of cardiac glycoside.

#### 2.5.6. Test for Steroids

Five (5) drops of concentrated H_2_SO_4_ were added to 1 ml of the extracts. Red coloration indicates the presence of steroids.

#### 2.5.7. Test for Phenolics

Two (2) drops of 5% FeCl_3_ were added to 1 ml of the extracts and the greenish precipitate indicates the presence of phenolics.

#### 2.5.8. Test for Cardenolides and Denolides

Exactly 2 ml of glacial acid containing one drop of 5% *w*/*v* FeCl_3_ was added to 1 ml of *F. exasperata* ethanol extract. 1 ml of concentrated H_2_SO_4_ was gently poured into the solution. A brown ring at the interface indicates the presence of cardenolides.

### 2.6. Proximate Analyses

The parameters determined for proximate analyses include ash, moisture, crude protein, fat, fiber, ether extract, and nitrogen-free extract. All of these were carried out using the methods described by [15].

### 2.7. Animal Treatments and Experimental Design

The experimental animals were divided into five groups of seven animals, each according to their body weight. Group I served as the control and received distilled water only. Group II rats received 250 mg/kg of APAP for 5 days. Group III, IV, and V served as test and were first given the ethanolic *F. exasperata* extract at concentration of 150, 250, and 500 mg/kg for 5 days, respectively, followed by a complementary administration of 250 mg/kg of APAP acetaminophen for another 5 days. At the end of the treatment, the rats were sacrificed, and the blood samples were collected in a clean dry heparinized bottle and allowed to clot. The serum was separated by centrifugation at 2500 rpm for 15 min. Subsequent analysis for various biochemical tests, i.e., ALT, AST, ALP, and bilirubin were carried out. The organs (liver and kidney) were also collected, homogenized and placed in 0.9% NaCl buffer solution for biochemical tests.

### 2.8. Acute Toxicity Tests of Ethanol Extract of *Ficus exasperata* on Albino Rats

Ethanol extract of *F. exasperata* was administered orally in doses of 250, 500, 1000, 1500, and 2000 mg/kg to the group of rats (*n* = 3), and the percentage mortality was recorded for 24 h. The rats were observed for any gross behavioral changes and hyperactivity, convulsions, urination, and defecation.

### 2.9. Determination of Oxidative Stress and Antioxidant Indices

The liver of each rat was removed, weighed, and washed with ice-cold saline and then homogenized in cold potassium phosphate buffer (0.05 M, pH 7.4). Subsequently, the homogenate was centrifuged at 10,000 xg for 15 min at 4°C, and the supernatant was used for determining the oxidant/antioxidant markers. Protein concentration was determined according to the method of Bradford [17] using bovine serum albumin as standard. Catalase (CAT) activity was determined using H_2_O_2_ as a substrate according to the method described by Clairborne [18]. GSH was evaluated according to the method described by Jollow et al. [19]. Lipid peroxidation was determined as malondialdehyde levels (MDA) according to the method described by Tahnteng and Agboola [20].

### 2.10. Concentrations of Proinflammatory Biomarkers

Nitric oxide (NO) level was determined by measuring the testicular nitrite content, the stable end-products of NO. Liver nitrite content was obtained using a sodium nitrite curve as standard and expressed as micromolar of nitrites per milligram of protein according to the method described by Green et al. [21]. Myeloperoxidase (MPO) activity was assayed according to the method described by Granell et al. [22]. MPO activity was expressed as micromolar of H_2_O_2_per minute per milligram of protein.

### 2.11. Histopathology of the Liver

The liver of each group was removed, completely immersed in Bouin's fixative, and processed for paraffin wax embedding. Homologous sampling was ensured by obtaining the uniformity of the transverse sections of the liver and testes of each specimen. Sections of 5 *μ*m thicknesses were cut on a rotary microtome (Leica, Germany), and the slides were stained with hematoxylin and eosin according to the method of Bancroft and Layton [23]. The slides were examined with a light microscope (Olympus CH Japan) for histological and histomorphometric studies. A micrometre was calibrated using a slide with a customized 2 mm ruler engraved on a coverslip (Zeiss) for the histomorphometric measurements. Twenty sections of seminiferous tubules (ST) that were oval or circular were randomly chosen and measured in each group—control and experimental. The intratubular (lumen) diameters and the thickness of the germinal epithelium were measured using the graticule with micrometre eyepiece 10x and objective 40x of the light microscope. The diameter of the lumen of each ST was measured across the minor and major axes, and the mean diameter was calculated, while the thickness of the germinal epithelium was measured from its base to its free surface at the same magnification. Photomicrographs were taken with Sony DSC-W 30 Cyber-shot (Japan). All slides were coded before examination with light microscope by investigators who were blinded to control and treatment groups.

### 2.12. Statistical Analysis

All results were presented as mean ± standard deviation (SD). Data were analysed by using Microsoft Excel 2007 (Redmond, Washington, USA) and Graph Pad Prism 5 software (Graph Pad Software Inc., USA). All the data of treatment groups were compared with the control group by using a one-way ANOVA followed by Dunnett's multiple comparison tests. In all the groups, differences were considered statistically significant among groups when *p* < 0.05.

## 3. Results

### 3.1. Phytochemical Screening

Table 1 shows the results obtained for the phytochemical screening of the plant extract featuring the presence of alkaloids, tannins, saponins, terpenoids, flavonoids, cardiac glycosides, steroids, and cardenolides while phenolics and anthraquinones were absent or in trace quantities.

### 3.2. Proximate Composition of *F. exasperata* Leaves

Proximate analysis of the *Ficus exasperata* is shown in Table 2. Our results show that the plant has a high nitrogen-free extract (34.62 ± 0.003) and ether extract (18.24 ± 0.01), moderate protein (13.55 ± 0.002) and ash (12.76 ± 0.002) content, and appreciably low but good moisture (10.65 ± 0.004) and fiber (10.18 ± 0.007).

### 3.3. Acute Toxicity Effect of Ethanol Extract of *Ficus exasperata* on Rats Not Treated with APAP

Table 3 shows the effect of various concentrations of *F. exasperata* extracts on daily behavior and mortality rate of rats. No mortality was recorded after 24 h; however, there was recorded a dose-dependent increase in severity of convulsion and urination.

### 3.4. Evaluation of Effect of *Ficus exasperata* Leaf Extracts on Liver Function Tests of APAP-Induced Liver Damage in Rats

Administration of acetaminophen (250 mg/kg) to rats caused significant (*p* < 0.05) elevation in AST, ALP, and AST enzyme levels and total bilirubin when compared to control. Pretreatment with *F. exasperata* leaf extract (150–500 mg/kg) restored these enzyme levels and that of total and direct bilirubin in extract-treated groups to levels comparable to the control. The decreases were found to be dose-dependent. This study was done in the liver and the serum as shown in Tables 4 and 5.

### 3.5. Effect of *Ficus exasperata* Leaf Extracts on Oxidative Stress and Antioxidant Markers in APAP-Induced Toxicity in the Liver

We assessed the level of oxidative stress and antioxidant markers in rats pretreated with *F. exasperata* extracts and thereafter administered acetaminophen (APAP) overdose. Our results revealed that APAP at dose 250 mg/kg b.wt significantly (*p* < 0.05) depleted glutathione (GSH, Figure 1(b)) level, decreased hepatic catalase (CAT, Figure 1(a)) activity with concomitant significant (*p* < 0.05) reduction in glutathione s-transferase (GST, Figure 1(c)), and superoxide dismutase (SOD, Figure 1(d)) activities, respectively, while it elevated nitric oxide (NO, Figure 2(a)) and lipid peroxidation (LPO, Figure 2(c)) levels when compared to control group. However, pretreatment with *F. exasperata* extracts at 150, 250, and 500 mg/kg. b.wt. significantly restored the levels and activities of NO, LPO GSH, CAT, GST, and SOD in dose-dependent manner when compared to APAP-control (*p* < 0.05).

### 3.6. Effect of *Ficus exasperata* Leaf Extracts on Inflammatory Markers in APAP-Induced Toxicity in the Liver

We assessed the level of inflammatory markers in rats pretreated with *F. exasperata* extracts and thereafter administered acetaminophen (APAP) overdose. Our results revealed that 250 mg/kg APAP significantly (*p* < 0.05) elevated iNOS (Figure 3(a)), COX-2 (Figure 3(b)), TNF-*α* (Figure 3(c)), IL-1*β* (Figure 3(d)), MCP-1 (Figure 3(e)), and IL-6 (Figure 3(f)) levels. However, pretreatment with *F. exasperata* extracts at 150, 250, and 500 mg/kg significantly restored activities of iNOS, COX-2, TNF-*α*, IL-1*β*, MCP-1, and IL-6 levels in dose-dependent manner when compared to the APAP-control (*p* < 0.05).

### 3.7. Effect of *Ficus exasperata* Leaf Extracts on Liver Histopathology in APAP-Induced Toxicity in the Liver

The photomicrographs of the histological structures of the liver are shown in Figure 4. Although the histology of the control group (A) shows no alteration, those of the APAP group (B) show visible lesions, while other groups did not show any visible lesions as compared to the control.

## 4. Discussion

Herbal-derived medicines are potential sources of bioactive compounds and phytocomponents that is involved in the scavenging of reactive oxygen species generated from toxic compound metabolism [24–26]. Broad ranges of pharmacological activities and responses have been reported for such compounds [16, 27]. The ability of natural compounds to attenuate toxin-induced hepatotoxicity is believed to be related to their intrinsic antioxidant properties [16]. Flavonoids and saponins, plant phytochemical constituent, are well known for their antioxidant and hepatoprotective activities [16]. The present study indicated that *F. exasperata* extracts are a dependable source of tannins, cardiac glycosides, proteins, and fiber. Batiha et al. [16] posit that flavonoids present in plants possess medical benefits including antioxidant and anti-inflammatory activities and have the ability to scavenge hydroxyl radicals, superoxide anions, and lipid peroxy radicals, thus bolstering its antioxidant activity. Accordingly, in our study, we detected the presence of flavonoids in *F. exasperata* extracts. Also, plant steroids have been shown to possess therapeutic applications as arrow poisons or cardiac drugs [28]. Thus, small quantities in plants would promote nitrogen retention and alleviate illness [29]. Plant steroids were also detected in *F. exasperata* extracts making it a suitable plant for drug-induced toxicity.

*F. exasperata* extracts were found to have high nitrogen-free extract (34.62 ± 0.003) and ether extract (18.24 ± 0.01), moderate protein (13.55 ± 0.002) and ash (12.76 ± 0.002) content, and appreciably low but good moisture (10.65 ± 0.004) and fiber (10.18 ± 0.007). Proteins play a significant role in body development, hormonal action, and enzyme activity [30]. Crude fiber content of *F. exasperata* extract may help gut health [31] and aid in the management of constipation problems [32]. Furthermore, the moderate ash content may clearly implicate in the treatment and management of drug-induced toxicity. Acetaminophen (APAP), a commonly used analgesic, and the antipyretic drug are metabolized by CYP450 enzymes to give N-acetyl-P benzoquinone-imine at extreme doses correspondingly causing covalent binding to thiol groups of reduced glutathione in the liver and kidney, depleting glutathione, and increasing the risk for hepatotoxicity [33].

Liver damage is characterized by elevated serum ALT, ALP, AST, and total bilirubin levels, which are biomarkers of liver functioning [34]. Our results show that APAP administration elevated the serum levels of ALT, ALP, AST, and total bilirubin, partly suggesting liver toxicity. However, on pretreatment with *F. exasperata* extracts restored the levels of these liver biomarkers to normal status compared to APAP group. These effects may be due to the potent antioxidant activity of alkaloids, flavonoids, tannins, steroids, and saponins isolated from the plant extract [35], which is likely to protect liver membranes from disruption. In addition to hepatic enzymes activity analysis, oxidative stress markers have also been described to demonstrate the involvement and occurrence of oxidative injury [36].

Glutathione (GSH/GSSG) is regarded as the main redox buffer in cells. Glutathione plays an important role in the removal of ROS and protects the thiols in biomacromolecules (SOD, CAT, GPx, and GR) [37], which maintain the prooxidant/antioxidant balance in the body [37]. To eliminate ROS from the cellular system, SOD and CAT function coordinately to remove superoxide radicals [38]. Particularly, lipid peroxidation disrupts cell membrane and function, resulting in tissue damage that weakens the antioxidant defense system needed to prevent ROS formation in APAP-intoxicated rats [39]. However, we observed an inhibition of lipid peroxidation as evidenced by reduced levels of MDA produced, thereby preserving the integrity of the rat's liver membrane. Similarly, pretreatment with extracts *F. exasperata* ameliorated APAP-induced depletion in GSH level, reduction in NO, LPO levels, and inhibition of CAT, SOD, and GST activities, respectively. Furthermore, APAP-induced hepatotoxicity led to significant increase in inflammatory proteins including iNOS, COX-2, IL-1*β*, IL-6, MCP-1, and NF-*κ*B; this is in line with several studies as reviewed by Egbuna [37]. IL-1*β* is increased early in acetaminophen toxicity and may be important in iNOS induction also monocyte chemoattractant protein-1 (MCP-1) and appears to be involved in hepatocyte repair and the regulation of proinflammatory cytokines [40]. However, EFE administration was able to counteract the effect of APAP in Wistar rat liver.

For the study of acute toxicity of the plant extract, it was found that the oral administrations of the ethanolic extract of *Ficus exasperata* up to 2000 mg/kg produced mild toxic effects in the normal behavior of the rats. However, no mortality was observed, and from this observation, it might be suggested that the plant to some extent is safe at this given doses. Ethanolic extract of *Ficus exasperata* did not show any toxicity and behavioral changes in rats up to 2000 mg/kg and might be considered to be safe as a herbal drug [41]. Although the phytoconstituents of *F. exasperata* may be responsible for its hepato-protective activity, necessary and detailed molecular studies should be carried out to elucidate the precise mechanisms of action of the phytoconstituents.

## 5. Conclusion

The data from this study suggest that ethanolic *F. exasperata* extract possesses antioxidant activity and can effectively protect against acetaminophen-induced oxidative stress and liver damage in Wistar rats. Increased levels of antioxidant enzymes and reduced oxidative stress products are strongly associated with *F. exasperata* extracts as an agent capable of alleviating hepatotoxicity caused by acetaminophen overdose. Thus, this study shows experimental proof and justifies the traditional claims and use of *F. exasperata* in treating liver dysfunction and diseases.

## Figures and Tables

**Figure 1:** Effect of *Ficus exasperata* leaf extracts on antioxidant markers in APAP-induced toxicity in the liver.

**Figure 2:** Effect of *Ficus exasperata* leaf extracts on antioxidant markers in APAP-induced toxicity in the liver.

**Figure 3:** Effect of *Ficus exasperata* leaf extracts on inflammatory markers in APAP-induced toxicity in the liver.

**Figure 4:** Photomicrographs of acetaminophen-induced toxicity in rat liver and treated with ethanolic extract of *Ficus exasperata*. (a) Control, (b) APAP only (250 mg/kg), (c) APAP +EFE (150 mg/kg), (d) APAP + EFE (250 mg/kg), (e) APAP + EFE (500 mg/kg). APAP: acetaminophen; EFE: ethanolic extract of *Ficus exasperata*; H & E 100x CV: central vein.

**Table 1:** Phytochemical screening of the ethanoic extract of leaf of *Ficus exasperata.*

Phytochemical component	Ethanol extracts
Saponin	+
Steroid	+
Phenolics	—
Cardenolides and denolides	+
Flavonoids	+
Tannin	+
Anthraquinone	—
Cardiac glycosides	+

+: detected; -: not detected.

**Table 2:** Proximate analysis of the ethanolic extract of *Ficus exasperata*.

Content (%)	Value (%)
Moisture	10.65 ± 0.004
Total ash	12.76 ± 0.002
Crude protein	13.55 ± 0.002
Crude fiber	10.18 ± 0.007
Ether extract	18.24 ± 0.010
Nitrogen free extract	34.62 ± 0.003

Results are expressed as mean ± standard deviation.

**Table 3:** Mortality rates and behavioral sign studies in rats given ethanolic extracts of *Ficus exasperata.*

Group	Dose (mg/kg)	Route	Behavioral signs	Mortality
1	250	Oral	Hyperactivity, convulsion, urination, and defecation	No death after 24 hours
2	500	Oral	Hyperactivity, defecation	No death after 24 hours
3	1000	Oral	Hyperactivity, convulsion, and urination	No death after 24 hours
4	1500	Oral	Convulsion, urination	No death after 24 hours
5	2000	Oral	Convulsion, salivation, and urination	No death after 24 hours

**Table 4:** Effect of *Ficus exasperata* leaf extracts on liver function enzymes in the serum of rats treated with APAP.

Groups	AST (U/L)	ALT (U/L)	ALP (U/L)	TOTAL BIL (U/L)
Control	15.14 ± 2.43	10.22 ± 1.47	201.33 ± 4.57	2.77 ± 0.54
APAP only (250 mg/kg)	56.31 ± 4.83^a^	37.74 ± 2.12^a^	111.37 ± 3.87^a^	5.86 ± 0.75^a^
APAP + EFE (150 mg/kg)	22.33 ± 2.48^a^	12.43 ± 3.11^a^	162.88 ± 5.31^a^	3.54 ± 0.33
APAP + EFE (250 mg/kg)	21.47 ± 1.33	16.77 ± 1.21	183.44 ± 6.22	3.61 ± 0.64^a^
APAP + EFE (500 mg/kg)	20.42 ± 3.58	14.73 ± 1.75^a^	147.32 ± 4.56^a^	3.79 ± 0.57

**Table 5:** Effect of *Ficus exasperata* leaf extracts on liver function enzymes in the liver of rats treated with APAP.

Groups	AST (U/L)	ALT (U/L)	ALP (U/L)	Total Bil (U/L)
Control	30.52 ± 5.30	34.29 ± 3.28	92.43 ± 5.55	1.11 ± 0.31
APAP only (250 mg/kg)	54.33 ± 2.13^a^	49.14 ± 3.52^a^	240.33 ± 7.97^a^	5.60 ± 0.57^a^
APAP + EFE (150 mg/kg)	32.44 ± 3.14	35.03 ± 2.87^a^	113.42 ± 6.21^a^	2.16 ± 0.42
APAP + EFE (250 mg/kg)	36.49 ± 3.17	33.22 ± 3.11^a^	141.34 ± 5.21	2.45 ± 0.49^a^
APAP + EFE (500 mg/kg)	33.12 ± 2.32^a^	31.21 ± 1.54	133.41 ± 5.64^a^	2.37 ± 0.31
